The article "High failure rate after Beta-tricalcium phosphate grafting for the treatment of femoral head osteonecrosis: a retrospective analysis" was retracted in 2021. Reason: lack of ethics approval or compliance.

# High failure rate after Beta-tricalcium phosphate grafting for the treatment of femoral head osteonecrosis: a retrospective analysis

**DOI:** 10.1186/s12891-020-03291-5

**Published:** 2020-04-27

**Authors:** Pei Liu, Xiao-hong Mu, Hua-chen Yu, Jian-lei Guan, Zhao-hui Liu, Wei-guo Wang, Qi-dong Zhang, Wan-shou Guo

**Affiliations:** 1 Beijing University of Chinese Medicine, Yinghuadong Road, Chaoyang District, Beijing, China; 2 Department Orthopedics 4, Beijing University of Chinese Medicine, Dongzhimen Hospital, Beijing, China; 3 Graduate School of Peking Union Medical College, Beijing, China; 4 Department of Orthopaedic Surgery, Beijing Key Lab Immune-Mediated Inflammatory Diseases, China-Japan Friendship Hospital, No. 2, Yinghuadong Road, Chaoyang District, Beijing, 100029 China

**Keywords:** Osteonecrosis of the femoral head, Beta-tricalcium phosphate, Head-preserving surgery

## Abstract

**Background:**

Non-vascularized bone grafting is a promising head-preserving technique for younger patients diagnosed as non-traumatic osteonecrosis of the femoral head (NONFH). Among the various types of bone grafting techniques, “light-bulb” procedure grafting with synthetic bone substitute is an attractive option. We aimed to assess the effectiveness of using beta-tricalcium phosphate (β-TCP) for the treatment of pre-collapse and early post-collapse lesions NONFH.

**Methods:**

From April 2010 to June 2014, 33 patients (47 hips) with NONFH were treated using the afore-mentioned technique. The clinical and radiological outcomes were recorded and compared statistically between pre- and post-operation. Harris hip score (HHS) was used to evaluate the clinical results, and Association Research Circulation Osseous (ARCO) stage was applied to assess the radiological outcomes.

**Results:**

The 5-years survival rate of using β-TCP grafting was accounting for 25.5%. HHS was decreased from 78.47 to 52.87 points, and a very significant worsening of radiological results were revealed (*P* <  0.05). Two hips collapsed more than 2 mm were awaiting for THA, and 33 of the 47 hips had converted to THAs in an average time to failure of 24.24 months postoperatively. Meanwhile, only 4 hips survived without collapse, and 8 hips collapsed less than 2 mm. After surgery, the time onset of head collapse was 3.65 months on average, and the first conversion to THA was performed at 5 months postoperative.

**Conclusions:**

Our results suggest that “light-bulb” procedure grafting with β-TCP sticks presented with a high failure rate in the early postoperative period. It is not proposed for the treatment of pre-collapse and early post-collapse lesions NONFH.

## Background

Non-traumatic osteonecrosis of femoral head (NONFH) is a devastating condition associated with apoptosis of the osteocytes and the bone marrow, which has a natural history of relentless progressive necrosis leading to fracture of subchondral bone plate, collapse of femoral head articular surface, and eventual premature osteoarthritis of hip [1, 2]. Meanwhile, NONFH is a challenging disease as it frequently disturbs young patients between second and fifth decades, the etiologies and risk factors are multiple, the pathogenesis is unknown, early diagnosis is difficult, and the successful treatment is undetermined [3]. Therapeutic methods have been developed for the treatment of NONFH can be assigned into three categories: non-surgical management, head-preserving surgery and hip-replacing procedures. Being a progressive disease, non-surgical management is generally unsuccessful. Total hip arthroplasty (THA) is also not a favorable treatment for young patients due to their long life expectancy. Therefore, many head-preserving procedures are proposed to protect the involved hip from collapse, which include a large single or multiple small holes core decompression (CD) [4, 5], osteotomies in various types [6, 7], and bone grafting in different methods [8, 9].

The article "High failure rate after Beta-tricalcium phosphate grafting for the treatment of femoral head osteonecrosis: a retrospective analysis" was retracted in 2021. Reason: lack of ethics approval or compliance.

The “light-bulb” technique initially described by Rosenwasser, in which a window is made at the femoral head neck junction, allows the debridement of necrotic tissue then subsequent bone grafting [10]. Donor bone tissues can be divided into autograft, allograft, and synthetic bone substitute. Autologous bone graft is considered as the gold standard, but it may require additional surgeries, and is related with donor-site complications [11]. Allograft is restrained by disease transmission, possible immune rejection, and lower incorporation rate compared to autograft [12]. Some synthetic bone substitutes through mimicking the structure, properties, and function of natural bone have been used as feasible alternatives to support the subchondral bone of femoral head, and to avoid donor-site morbidity [13]. Characterized by easy biodegradation and high osteoconduction [14], beta-tricalcium phosphate (β-TCP) is used to refill the bone defect and provide initial mechanical support for ONFH in clinical practice [15].

We hypothesized that “light-bulb” procedure grafting with β-TCP for the treatment of pre-collapse and early post-collapse lesions NONFH could alleviate pain, stimulate bone formation, support the subchondral bone and articular cartilage of femoral head, maintain a congruent hip, improve joint function, and if possible, defer or avert the requirement for THA. In this study, we report results of this management and clarify its value.

The article "High failure rate after Beta-tricalcium phosphate grafting for the treatment of femoral head osteonecrosis: a retrospective analysis" was retracted in 2021. Reason: lack of ethics approval or compliance.

## Patients and methods

This study was approved by the Ethics Committee of the China-Japan Friendship Hospital (2015-SFZX-N). We retrospectively reviewed all patients with symptomatic NONFH who underwent “light-bulb” procedure grafting with β-TCP sticks (Shanghai Bio-lu Biomaterials, Shanghai, China) in our institution between April 2010 and June 2014. We claimed no research fund to the present study from Bio-lu Biomaterials Co. Ltd.

The diagnosis of NONFH was drawn based on history, clinical symptoms, physical examination, related risk factors and imaging data. Necrotic lesions of the femoral head were graded according to the Association Research Circulation Osseous (ARCO) stage [16]. Patients who presented with NONFH in ARCO stage II or IIIa were included for the proposed procedure [8], and exclusion criteria were: (1) over-aged, mainly above 50 years; (2) unable to stop corticosteroids administration due to corticosteroid-dependent diseases; (3) failed to quit alcohol abuse. Patients who were in ARCO stage IV or in ARCO stage IIIb and IIIc with complaints of serious pain were included for THA [17].

Demographic patient data were collected from our hospital medical registry. In total, 37 patients with NONFH were treated with the recommended technique, and 4 of these patients were lost to follow-up. Finally, 33 patients (47 hips; 6 in female), with a mean age of 36.3 ± 8.0 years (range 23 years to 49 years) at the time of surgery were included. The risk factors included excessive intake of alcohol (consuming > 400 mL weekly) in 11 patients (17 hips), corticosteroids (2 g or more of systemic corticosteroids administered over a 3-month period minimum) in 19 patients (26 hips), and idiopathic in 3 patients (4 hips). Detailed information can be seen in Table 1, and the study conforms to the STROBE (strengthening the reporting of observational studies in epidemiology) statement (Fig. 1).

**Table 1:** Demographic characteristics of patients with NONFH

Total patient number	47 hips (33 patients)
Mean age at surgery	36 years (23–49 years)
Gender ratio	Male/Female = 27/6
Involved hip	Unilateral/Bilateral = 19/14
Risk factors	
Corticosteroid	19 patients (26 hips)
Alcoholism	11 patients (17 hips)
Idiopathic	3 patients (4 hips)

**Fig. 1:** Flowchart of the study

After anesthesia, patient laid in the supine position. The direct anterior approach (DAA) was taken to expose the anterolateral femoral head-neck junction. And then, osteotomies were used to create a bone window (1.5 cm in width and length). With the aid of C-arm fluoroscopy images, the necrotic tissue was debrided using bone drills and curettes. A minimum of 5 mm subchondral bone was kept. A number of holes were made using a 3.2 mm drill to the extent that the surface of the sclerotic bone was observed to bleed. After debridement, the cavity was cleared by irrigation. The β-TCP sticks were impacted in layers. The original resected bone plate was grafted into the bone window without being fixed. Thorough sterilization with saline solution was carried out to prevent heterotopic ossification of the surgical site before the incision was closed.

The article "High failure rate after Beta-tricalcium phosphate grafting for the treatment of femoral head osteonecrosis: a retrospective analysis" was retracted in 2021. Reason: lack of ethics approval or compliance.

All patients received a strict post-operative rehabilitation plan under the guidance of an experienced doctor (Wei-guo Wang). Patients were instructed to do isometric quadriceps exercise immediately after the operation. It was advised to practice toe-touching exercises in the course of first 3 months, and gradual weight-bearing was allowed for the subsequent 3 months with the aid of a cane or crutch on the opposite side. Patients began full weight-bearing in the 6th month after surgery. From the 12th post-operative month, patients were permitted to engage in high impact activities (such as running).

After surgery, clinical and radiological follow-up of all cases was conducted by the researchers of this study at the interval of 3 months in the first year and 6 months in the subsequent years. The clinical follow-up examined pain, function, deformity, and range of motion based on pre- and post-operative Harris Hip Score (HHS) difference [18]. The radiological follow-up consisted of radiographs taken at each visit from the antero-posterior and frog-leg lateral views of the bilateral hips. Clinical failure was defined as HHS ≤ 70 points or conversion to THA for any reason. Radiographic failure was defined as the collapse > 2 mm or premature osteoarthritis according to follow-up radiographs. The time-to-failure was calculated as the time between the date of surgery and the date of clinical failure or radiographic failure. The onset time of head collapse was defined as the earliest period between the date of surgery and the date of follow-up discovering collapse progression.

The SPSS package for Windows (Version 20.0; SPSS Inc., Chicago, Illinois, USA) was applied for statistical analysis. The continuous variable was expressed as the mean ± standard deviation. The Kolmogorov-Smirnov test was used to confirm the normality of the measured data. Wilcoxon test was performed to assess differences in HHS between pre- and post-operation. *P* <  0.05 was considered to have statistical significance.

## Results

We followed up with the patients that didn’t undergo THA for a minimum period of 5 years, and the mean follow-up was 36.09 ± 22.08 months (range 5 months to 75 months) for all 47 hips (Table 2). No perioperative complications were detected.

The article "High failure rate after Beta-tricalcium phosphate grafting for the treatment of femoral head osteonecrosis: a retrospective analysis" was retracted in 2021. Reason: lack of ethics approval or compliance.

**Table 2:** Outcomes of patients treated with β-TCP grafting

Case	Gender/Age	Etiology	Laterality	Preoperative			Follow-up				Outcomes
				ARCO stage	HHS	HPS	ARCO stage	HHS	HPS	Survival (months)	
1	M/26	Alcoholism	Right	IIc	80	30	IIc	80	40	75	No progression
			Left	IIIa	75	20	IIIc	45	10	22	THA
2	F/39	Corticosteroid	Right	IIc	86	30	IIIa	70	20	62	Collapse ≤2 mm
			Left	IIIa	73	20	IV	34	10	10	THA
3	M/42	Alcoholism	Left	IIIa	74	20	IV	42	10	22	THA
4	M/46	Alcoholism	Right	IIc	80	30	IIIa	75	20	60	Collapse ≤2 mm
			Left	IIIa	72	20	IV	34	10	12	THA
5	M/44	Alcoholism	Right	IIc	86	30	IV	48	10	23	THA
			Left	IIIa	75	20	IV	45	10	48	THA
6	M/23	Corticosteroid	Right	IIc	85	30	IV	40	10	12	THA
			Left	IIb	90	44	IV	64	20	12	THA
7	F/34	Corticosteroid	Right	IIIa	70	20	IV	41	10	21	THA
8	M/31	Corticosteroid	Right	IIc	78	30	IIIc	64	10	23	THA
			Left	IIb	90	40	IV	61	20	23	THA
9	M/42	Corticosteroid	Right	IIc	75	30	IV	40	10	12	THA
			Left	IIb	90	40	IIIc	59	10	5	THA
10	M/33	Corticosteroid	Right	IIc	79	30	IIc	80	30	68	No progression
			Left	IIb	86	30	IIb	84	30	68	No progression
11	M/37	Corticosteroid	Left	IIc	79	30	IIIa	80	20	75	Collapse ≤2 mm
12	M/32	Alcoholism	Right	IIc	83	30	IIIa	78	20	66	Collapse ≤2 mm
			Left	IIc	86	30	IIIa	80	20	66	Collapse ≤2 mm
13	M/42	Corticosteroid	Right	IIIa	75	20	IIIc	39	10	22	THA
14	M/27	Corticosteroid	Right	IIc	80	30	IIIa	79	20	69	Collapse ≤2 mm
15	F/49	Idiopathic	Right	IIIa	70	20	IV	40	10	36	THA
			Left	IIIa	72	20	IV	44	10	36	THA
16	F/35	Corticosteroid	Left	IIIa	75	20	IIIc	50	10	23	THA
17	M/49	Corticosteroid	Left	IIIa	70	30	IIIc	42	10	35	THA
18	M/46	Alcoholism	Right	IIc	84	30	IV	38	10	24	THA
			Left	IIIa	70	20	IV	45	10	11	THA
19	M/24	Idiopathic	Right	IIb	84	30	IIIa	75	30	72	Collapse ≤2 mm
20	M/42	Corticosteroid	Left	IIIa	74	20	IV	39	10	56	THA
21	M/40	Alcoholism	Left	IIc	79	30	IV	40	10	12	THA
22	M/35	Alcoholism	Left	IIIa	72	20	IIIc	49	10	45	THA
23	M/27	Corticosteroid	Left	IIIa	75	20	IIIa	70	20	68	No progression
24	M/24	Corticosteroid	Right	IIIa	76	20	IIIb	58	20	60	Advanced collapse
			Left	IIIa	69	20	IIIb	53	20	66	Advanced collapse
25	M/28	Idiopathic	Left	IIb	88	40	IIIa	75	20	70	Collapse ≤2 mm
26	M/34	Alcoholism	Left	IIIa	75	20	IIIc	45	10	50	THA
27	M/45	Corticosteroid	Left	IIIa	75	20	IV	35	10	22	THA
28	M/41	Alcoholism	Right	IIIa	70	20	IIIc	40	10	40	THA
29	M/49	Corticosteroid	Left	IIIa	76	20	IV	38	10	12	THA
30	F/31	Corticosteroid	Left	IIIa	71	20	IIIc	45	10	11	THA
31	F/24	Corticosteroid	Right	IIIa	76	20	IIIc	40	10	11	THA
			Left	IIc	81	30	IV	37	10	16	THA
32	M/44	Corticosteroid	Left	IIb	86	40	IV	42	10	9	THA
33	M/35	Alcoholism	Right	IIb	90	40	IV	38	10	24	THA
			Left	IIc	86	40	IV	45	10	9	THA

Preoperative HHS was 78.47 ± 6.39 points, and it was 52.87 ± 16.14 points at the final follow-up, indicating that clinical functions became poorer (*P* <  0.05) (Table 3). When checking the four elements (pain, function, deformity, and range of motion) in the scale of HHS pre- and post-operatively, we found that the reduction of Harris pain score (HPS) was the heaviest contributor to general degradation of HHS. It was changed from 38.00 to 18.75 points in ARCO IIb hips, 30.63 to 16.88 points in ARCO IIc hips, and 20.43 to 11.30 points in ARCO IIIa hips (*P* <  0.05).

The article "High failure rate after Beta-tricalcium phosphate grafting for the treatment of femoral head osteonecrosis: a retrospective analysis" was retracted in 2021. Reason: lack of ethics approval or compliance.

**Table 3:** Comparison of pre- and post-operative HHS, HPS

ARCO stage	Hips	Pre-operation		Post-operation		*P* value HHS/HPS
		HHS	HPS	HHS	HPS	
IIb	8	87.87 ± 2.03	38.00 ± 5.13	62.25 ± 16.09	18.75 ± 8.35	0.004/0.003
IIc	16	81.50 ± 3.61	30.63 ± 2.50	60.88 ± 18.61	16.88 ± 8.73	0.001/< 0.001
IIIa	23	73.09 ± 2.45	20.43 ± 2.09	44.04 ± 8.12	11.30 ± 3.44	< 0.001/< 0.001
Total	47	78.47 ± 6.39	26.89 ± 7.43	52.87 ± 16.14	14.47 ± 7.17	< 0.001/< 0.001

On radiographs, a very significant worsening was revealed in all stages (*P* <  0.05) (Table 4). Only 4 hips (8.5%) survived without further collapse, and collapse of the femoral head ≤2 mm was observed in 8 hips (17.0%) during 5-year follow-up. Meanwhile, 2 hips collapsed > 2 mm were awaiting for THA, 33 of 47 hips had converted to THAs in an average time-to-failure of 24.24 ± 14.39 months postoperatively. Gradual biodegradation of the β-TCP sticks without new bone formation was noted in the early postoperative period (Fig. 2). The average onset time of head collapse was 5.58 ± 2.69 months (range 1 month to 12 months) after surgery, and the 2-year failure rate of head-preserving was 75.8% (25/33) (Fig. 3). Among the hips converted to THAs, no complications occurred due to minimally invasive surgery. The resected femoral heads were sent for further examination. Gross examination showed the grafting bone substitute was muddy, and microscopic examination displayed only fibrotic and necrotic tissues in the femoral head without signs of new bone were observed (Fig. 4).

**Table 4:** Comparison of pre- and post-operative values in different AROC stages

ARCO stage	Before operation (hips)	At last follow-up (hips)	*P* value
IIb	8	1	0.03
IIc	16	2	0.01
IIIa	23	9	0.02
IIIb, IIIc, and IV	0	35	< 0.001

**Fig. 2:** A 24 year-old female patient (case 31): **a**-**c** Preoperative radiographs showed bilateral NONFH with right ARCO IIIa stage and left ARCO IIc stage. **d**-**f** Postoperative imaging at 1 week exhibited adequate filling of the osteonecrotic lesion by the beta-tricalcium phosphate (β-TCP). **g**-**i** At 8 weeks, the right head presented advanced collapse, and the β-TCP were gradually absorbed. Also, heterotopic ossification was observed in right side. **j**-**l** At 20 weeks, the right femoral head collapsed more than 4 mm and the contralateral collapsed less than 2 mm. In the meantime, the sparse remnants of grafting materials were almost entirely degraded

**Fig. 3:** Failure rate of head-preserving using β-TCP grafting

**Fig. 4:** β-TCP in the grafting area was muddy, and only fibrotic and necrotic tissues in the femoral head without signs of new bone were observed

The article "High failure rate after Beta-tricalcium phosphate grafting for the treatment of femoral head osteonecrosis: a retrospective analysis" was retracted in 2021. Reason: lack of ethics approval or compliance.

## Discussion

The most important finding of this study was that “light-bulb” procedure grafting with β-TCP sticks was associated with a high failure rate for the treatment of pre-collapse and early post-collapse lesions NONFH. To our knowledge, this study is the first to report the poor results in the early postoperative period.

Generally, a genetic predisposition and exposure to risk factors exert a synergistic effect in the NONFH pathogenesis [19]. The impaired blood supply to the femoral head results in cellular apoptosis, subchondral fracture, and collapse at a later stage, subsequently deteriorate disabled osteoarthritis. Most authors believe that effective intervention at an early stage can successfully protect these hips from collapse [20]. The “light-bulb” technique obtains outstanding clinical efficacy, at a mean follow-up of 12 years, showing success in 84.6% (11) of 13 hips [10]. The success of this technique depends on replacing the necrotic segment with cortical bone graft plus fresh cancellous, achieving intra-osseous decompression of the necrotic segment, and providing adequate structural support in order to allow subchondral bone plate remodeling and healing. Mont et al. reported the utilization of bone morphogenetic protein-enriched allograft through the treatment with an 86% success rate after a mean of 48-months follow-up [21]. Another review of the “light-bulb” procedure using auto-iliac bone combination of demineralized bone matrix, at a mean follow-up of 25 months, stated 68% survivorship of 138 hips in early and medial stages of ONFH [22]. We detailed a similar procedure in which the necrotic bone was debrided through DAA and replaced by β-TCP sticks. We tended to determine whether a similar or high success rate could be obtained by using synthetic bone graft substitutes that avoided donor site morbidity.

Things turn out to be worse than we imagined. In this study, there was a high failure rate (74.5%) on using β-TCP with advanced collapse and converting to THA. At 5 years of follow-up, the survivorship was 25.5%, with 4 hips surviving without collapse of the femoral head and 8 hips collapse less than 2 mm. The onset of head collapse was 3.6 months on average, and the first conversion to THA was performed at 5 months postoperative. From the appearance, the β-TCP grafts looked softened and muddy structure without new bone formation, when the specimens harvesting from the resected femoral head during THA.

β-TCP is a class of tunable calcium phosphate that has been widely used for bone grafting because of its excellent reliability, biocompatibility, and osteoconductive properties [23]. When employed for the treatment of NONFH, it may be a promising bioactive material because it can fill up the necrotic lesion, be degraded gradually by creeping substitution, and act as a scaffold for the repair of the osteonecrotic femoral head. In this study, it failed to treat NONFH successfully because of biodegradation immediately and lack of vascularization.

The article "High failure rate after Beta-tricalcium phosphate grafting for the treatment of femoral head osteonecrosis: a retrospective analysis" was retracted in 2021. Reason: lack of ethics approval or compliance.

The β-TCP may have enough mechanical strength initially, but loses its structural support latterly due to degrade early after implantation. After removing the necrotic lesion, a bone cavity is produced in the femoral head. Theoretically, the degradation of bone grafts should be synchronized with the formation of new bone. The total biodegradation of β-TCP lasted over 12 weeks in a contained osseous defect [24]. During the process, a series of reactions including vascular infiltration, osteoid deposition, and restoration of the defect with new mineralized bone trabeculae occurred successively. A pilot study performed by Rijnen et al. showed that the absorption process of calcium phosphate cement took place in 6 weeks and was entirely completed in 12 weeks postoperatively [25]. Accelerated degradation leads to a rapid decrease of biomechanical strength in the necrotic site. As a result, these areas are prone to mechanical failure and fracture when stressed. A clinical trial conducted by Tomoki Aoyama et al. stated that the collapse of the femoral head was ascribed to the imbalance between the faster degradation of β-TCP and the weaker ability of osteogenesis [26].

Another possible reason is that the osteonecrotic environment in the femoral head is unfit for the β-TCP to repair the lesion. The vascular network is able to supply nutrients and remove waste products. Unlike autogenous bone tissues containing a highly vascularized network, current synthetic bone substitutes lack of vascularization, causing failure of the survivorship and function during the early phase of implantation [27]. There is accumulating evidence that the vascularized bone-grafting is crucial in the bone remodeling process [28]. Once a well-formed and stable small blood vessels incorporating into synthetic bone substitutes, the formation of new bone would be accelerated [29]. On the contrary, if the blood supply does not recover in time, β-TCP might undergo the necrotic process before integrating into the host body due to lack of nutrients and oxygen available within the constructs [30]. In a study of 19 hips managed with non-vascularized bone-grafting using injectable synthetic bone graft substitutes through a core track for the treatment of ONFH (ARCO IIC and IIIA), survivorship was 10.5% in the 5-year follow-up [31]. By contrast, vascularized bone grafting has resulted in excellent outcomes that many studies reported a 5 years survivorship was approximately 80% [32]. In a study on β-TCP granules mixed with vascularized iliac bone graft cultured with mesenchymal stem cells in 9 hips, 7 patients had no evidence of progression at a mean follow-up of 24 months [26]. Additionally, β-TCP lacks biological stimulatory activity [33]. All these factors indicate that β-TCP is not an optimal biomaterial to be applied in the treatment of NONFH.

The article "High failure rate after Beta-tricalcium phosphate grafting for the treatment of femoral head osteonecrosis: a retrospective analysis" was retracted in 2021. Reason: lack of ethics approval or compliance.

The limitations of this study include a small sample size without controls and its non-randomized study design. Whether the use of the β-TCP or other synthetic materials grafting is effective in other cases of NONFH cannot be answered by this study. Because of the poor results, we discontinued to recommend our patients on using light-bulb procedure combined with β-TCP sticks grafting in the treatment of NONFH. Further larger prospective random control trials are required to better validate our findings. Evaluation of magnetic resonance imaging, arthroscopic assessment of regenerated cartilage, and histological evaluation should be performed for all subjects at a certain period after surgery. Additionally, new tissue scaffolds such as bone graft substitutes combined with growth factors, and pre-vascularization bio-engineered bone may increase the survivorship of bone grafting [34].

## Conclusions

Treatment of NONFH with “light-bulb” and β-TCP sticks did not avoid or forestall the need for hip replacement. Therefore, it is not proposed for the treatment of pre-collapse and early post-collapse lesions NONFH.

## Data Availability

The datasets used and/or analyzed during the current study are available from the corresponding author on reasonable request.

## Abbreviations

ARCO: Association Research Circulation Osseous
β-TCP: Beta-tricalcium phosphate
CD: Core decompression
DAA: Direct anterior approach
HHS: Harris Hip Score
NONFH: Non-traumatic osteonecrosis of femoral head
THA: Total hip arthroplasty
